# Exploring the Risk Factors of Conjunctival Squamous Cell Carcinoma and Establishing a Prognostic Model: Retrospective Study

**DOI:** 10.1155/2022/5427579

**Published:** 2022-10-15

**Authors:** Bihua Xie, Zejun Chen, Jun Luo, Yanan Lei, Jiaojiao Li, Rongrong Wu, Quanting Wang, Xianan Liu

**Affiliations:** ^1^Department of Ophthalmology, Chengdu First People's Hospital, Sichuan Province, 610041, China; ^2^Department of Nephrology, Chengdu First People's Hospital, Sichuan Province, 610041, China; ^3^Department of Cardiology, Chengdu First People's Hospital, Sichuan Province, 610041, China

## Abstract

**Objective:**

Exploring the risk factors of conjunctival squamous cell carcinoma (CSCC) and establishing a prognostic model.

**Methods:**

Information on patients with CSCC was extracted from the SEER database, conducting a retrospective study. 650 patients with CSCC were finally included in the model. Descriptive analysis was performed by Chi-square test and *T*-test. The risk factors of CSCC were explored by COX multivariate analysis, and the corresponding prognostic model was established as a result.

**Results:**

The all-cause mortality rate of CSCC was 38.3%, and the risk factors were age (HR = 1.077), sex (HR = 0.691), grade (HR = 7.857), laterality (HR = 1.403), N (HR = 7.195), M (HR = 0.217), and surgery (HR = 1.618), all *P* < 0.05. The new model had C index and area under curve ROC (AUC) value greater than 0.7. Calibration curve, Net Reclassification Index (NRI), Integrated Discrimination Improvement (IDI), and Decision Curve Analysis (DCA) indicate the new model has better predictive performance than the American Joint Committee on Cancer (AJCC-TNM).

**Conclusions:**

Compared with the clinical guidance of AJCC (TNM) for patients with CSCC, the established model exhibits good performance and can provide guidance for clinical decision-making.

## 1. Introduction

Squamous cell carcinoma is a malignant tumor that easily occurs in various epithelial tissues. The ocular surface (conjunctiva and corneoscleral limbus) is one of the tissues prone to squamous cell carcinoma. It most frequently occurs at the corneoscleral limbus and exposed areas of bulbar conjunctiva. The conjunctiva is composed of nonkeratinized epithelial composition, including stratified squamous epithelium and stratified columnar, and is scattered with goblet cells [1]. The margin of the cornea and sclera is transformed from conjunctival epithelium to corneal epithelium, and the cell proliferation is more active, which is the predilection site of conjunctival squamous cell carcinoma. Conjunctival squamous cell carcinoma (CSCC) is a rare tumor but the most common among ocular surface nonpigmented malignant tumors [2]. Although reports on CSCC incidence vary worldwide, two disease patterns have been recognized [3]. The first pattern occurs in countries close to the equator where young men and women are equally affected and the disease is associated with human immunodeficiency virus (HIV) infection. The estimated incidence in these regions is 1.8 cases per 100,000 people per year [4]. The second type is observed in the elderly living in northern high latitudes, mainly affecting males (5 times that of females), and has nothing to do with HIV infection. For this pattern, the reported incidence of cancer is 0.03 to 0.84 per 100,000 people per year [5].

CSCC is the terminal stage of a series of diseases called ocular surface squamous cell tumors [6]. This illness has many clinical manifestations, and the most common symptoms are red eyes, photophobia, irritation, foreign body sensation, and white, painless, progressive growth on the eye surface [7]. Although CSSC is a potentially curable cancer, misdiagnosis will result in loss of treatment time, and in the worst case, the disease will progress to a life-threatening state [8]. At present, surgical resection under the microscope is the most commonly used technique. Only small lesions can be completely removed (Figure 1), and large lesions involving the orbit may require orbital exenteration (Figure 1). This radical technique includes the removal of all orbital contents including the periosteum [6]. Despite the available treatments, CSCC still has a high recurrence rate (up to 43%), and the cosmetic effect of the advanced disease remains poor [9] bringing trouble to the patient's postoperative life [10]. Therefore, a comprehensive and in-depth study of CSCC must be conducted.

The American Joint Committee on Cancer (AJCC, 8th edition) recently reviewed the classification of conjunctival squamous tumors. The clinical staging for carcinoma of the conjunctiva is based on tumor size with T as carcinoma in situ; T1 and T2 as tumor less than and more than 5 mm with breach in continuity of basement membrane, respectively; T3 as tumor invasion into adjacent tissues (excluding orbit); T4 as tumor invasion into surrounding tissues including orbit. [11]. AJCC (TNM) is currently the priority reference guide for cancer treatment. However, TNM as the main indication has been proven to have poor predictive capacity in forecasting all-cause mortality from CSCC in prior studies [12]. Bellerive et al. also showed that AJCC (TNM) has nothing to do with the initial clinical treatment of conjunctival cancer and proposed that the AJCC T3 category should be reviewed to distinguish diffuse SCC from extensive surface extension from tumors with deep scleral infiltration [12].

This study aims to explore the risk factors of CSCC based on patient information from the disease epidemic database Surveillance, Epidemiology, and End Results (SEER) and establish the corresponding prognostic model as a reference for clinical decision-making. The database is open to scholars free of charge, and we have obtained access to the data with the account number 11215-Nov2020.

## 2. Material and Methods

### 2.1. Data Sources

Data were obtained from the SEER database, one of the most representative large-scale tumor registration databases in North America that records information about the morbidity and mortality of millions of patients with cancer in some states and counties of the United States. This is a retrospective study, and patient consent for the data obtained from the SEER database was not necessary because no information that can be used to identify individual patients was extracted [13]. This research project was verified with and exempted by the review committee of Chengdu First People's Hospital. This report of the study is in accordance with the STROBE guidelines for observational studies. [14]. C69.0-conjunctiva was selected in the anatomical degree point of the database [Primary Site–labeled], followed by squamous cell carcinoma in the morphology option [ICD-O-3 Hist/behav, malignant], including 8050/3, 8051/3, 8052/3, 8070/3, 8071/3, 8072/3, 8073/3, 8074/3, 8075/3, 8076/3, 8083/3, 8084/3, 8094/3, and 8560/3. Information including age, sex, race, grade, laterality, combined summary stage, derived American Joint Committee on Cancer (AJCC) T, derived AJCC N, derived AJCC M, surgery, survival months, and status (living or dead) were also obtained. In the initial extraction of data from 988 patients with CSCC, 337 patients with missing values of T, N, and M and 1 outlier were excluded. Finally, 650 patients were included. The outcome is the CSCC patients' all-cause death due to any cause.

### 2.2. Data Analysis

Among the patients, 80% (*N* = 520) were randomly divided into the training cohort, and 20% (*N* = 130 cases) were divided into testing cohort. First, a descriptive analysis was performed on the data. Continuous variables were described by median quarterback interval values, categorical variables were expressed as percentages, and *P* values were obtained by *T*-test and Chi-square test. The training set was used in COX survival analysis to obtain the different variables of HR and further analyze the effect of different variables on patient survival outcomes. All variables influencing the final outcome of CSCC were incorporated into the model to establish its nomogram to predict the patient survival rates at 3, 5, and 8 years and compare the newly established model with the TNM model. C index and the area under the ROC curve (AUC) were applied to judge the discrimination of the model [15]. A calibration curve was employed to determine the calibration degree of the model [16]. NRI and IDI values were utilized to examine the consistency of the model's survival prediction with the actual situation [17, 18]. DCA curve was used to judge the clinical profitability of the model [19]. All data analyses were based on EXCEL (version 2019; http://www.microsoft.com) and R (version 4.0.3; http://www.r-project.org). A bilateral probability value of *P* < 0.05 indicated statistical significance. The research flow chart is shown in Figure 2.

## 3. Results

In the initial extraction of data from 988 patients with CSCC, 337 patients with missing values of T, N, and M and 1 outlier were excluded. Finally, 650 patients were included. The outcome was the CSCC patients' all-cause death due to any cause. A total of 650 patients were included, and 249 deaths were recorded. The all-cause mortality rate was 38.3%. The characteristics of the patients are shown in Table 1. In both the training and test sets, the median age of surviving patients was 62 years, while the median age of dying patients was 77 years. Men accounted for 73.8% of patient population and dominated the death cases accounting for almost 80%. Half of the grade records of patients were nearly unknown (53.5%), but do not qualify as missing value. AJCC (TNM) system codes the extent of the primary tumor (T), regional lymph nodes (N), and distant metastases (M), TX, N2, and M0 accounted for the largest proportion of patients in TNM staging. Most patients chose surgery. White patients were the most common (87.8%), which is consistent with the ethnic distribution in the United States.

### 3.1. Multifactor COX Analysis Results

The results of COX multivariate analysis are in Table 2, which revealed that stage, T, and race had no significant effect on the prognostic outcome of patients with CSCC (*P* > 0.05). Age was a risk factor, that is, prognosis worsens with age (*P* < 0.001). The female gender is a protective factor. The risk for women was 0.691 times that for men (*P* = 0.046). The number of grade IV tumors was 7.857 times higher than that of grade I (*P* = 0.01). The prognosis of tumors in the left eye was not as good as that in the right eye. N2 had 7.195 times the risk of N1 (*P* = 0.011), and M0 had 0.217 times the risk of MX (*P* = 0.044). The number of patients without surgery and missing records was 1,618 times greater than the number of patients undergoing surgery. Once conjunctival squamous cell carcinoma is diagnosed, especially when the tumor tissue in the early stage is limited and has not invaded into adjacent tissues, surgical resection should be selected as soon as possible. So far, surgery is still considered as a protective treatment measure for patients, which also provides tissue for diagnosis.

### 3.2. Establishment and Verification of Nomogram

According to the results of the COX multicause analysis, a nomogram was created for the seven variables that influence the prognostic outcome of CSCC: age, sex, grade, laterality, N, M, and surgery. After modeling, the C index was calculated for the new model and the TNM model. The training set C index of the new model was 0.744, while the test set was 0.716. This result demonstrated that the model had a high level of discrimination. On the contrary, the C index of the training set of the TNM model was 0.554, while the test set was 0.504. Therefore, this model does not show a good degree of discrimination, which is similar to a previous study [12]. These risk factors were integrated to establish a nomogram shown in Figure 3. In this nomogram, N staging had the greatest effect on prognosis, while laterality had the least impact on the survival rate of patients with CSCC.

The AUC values of the new model and TNM were also computed. As shown in Figure 4, the AUC values of the new model training set were 0.773, 0.777, and 0.781 for 3, 5, and 8 years, respectively, and those for the test set were 0.772, 0.771, and 0.746, respectively. The AUC values of the 3, 5, and 8 years of the TNM model training set were 0.532, 0.507, and 0.491, and the test set were 0.522, 0.507, and 0.491, respectively. These findings also suggest that the discrimination of the new model is superior to the TNM model.

A calibration curve was utilized to check the calibration performance of the model. As shown in Figure 5, the red diagonal dashed line was the standard line of the model. The four prediction points of the new model were all around the standard line, thus proving that it has good calibration performance. The NRI value of the new model was also calculated. The NRI values of the training set for 3, 5, and 8 years were 0.651 (0.404–0.934), 0.768 (0.518–0.953), and 0.802 (0.300–1.021), respectively, and those of the test set were 0.629 (0.142–1.025), 0.771 (0.328–1.101), and 0.675 (0.312–1.206), respectively. The IDI values of the model training set for 3, 5, and 8 years were 0.122, 0.209, and 0.263, and those of the test set were 0.095, 0.175, and 0.226, respectively (*P* < 0.001). The statistical results of NRI and IDI in Table 3 revealed that the new model was positively improved. Finally, the DCA curve of the model was drawn, as shown in Figure 6. The solid red line in the figure represents the newly established model, and the cyan dotted line represents the TNM model. The AUC of the new model was larger than that of the TNM model, indicating that the former has a greater clinical decision-making benefit than the latter.

## 4. Discussion

CSCC is the most common tumor of the conjunctival epithelium that is associated with the risk of permanent visual impairment. What is more, it has the ability to relapse, metastasize, and cause death [20]. It is thought CSCC is formed when abnormal cells pass through the basement membrane and enter the conjunctiva. In intraepithelial neoplasia (CIN), malignant cells are confined to the surface epithelium. The research shows that CSCC can enter the anterior chamber of the eye through the cornea and sclera. Besides, it also can enter the orbital septum and invade the soft tissues of the orbit, sinuses, and brain [21, 22]. These tumors may metastasize through lymphatic vessels or blood during the course of the disease. Owing to its significant potential to invade, CSCC is a high risk factor that endangers vision and life [22, 23]. For every 10° decrease in latitude, the incidence of CSCC increases by 49%. Since the beginning of the AIDS epidemic, the incidence of CSCC in Africa has been on the rise. When an individual is infected with HIV, the risk of developing CSCC increases by 12 times, despite the fact that UV exposure is rather steady [24, 25]. The harm of CSCC to people is evident. Hence, this study explored the risk factors of CSCC and established a corresponding prognostic model.

The AJCC (TNM) treatment guidelines for conjunctival cancer have been deemed inaccurate, which is in agreement with the findings of this study. The TNM model was utilized as the primary indicator to predict the long- and short-term survival of patients with CSCC. However, the survival rate effect is extremely poor, the C index and AUC values are extremely low, and no good degree of discrimination has been achieved. The proposed model shows outstanding discrimination (C index and AUC), calibration (calibration curve), model improvement (NRI and IDI), and clinical decision benefit (DCA) performance.

According to the established nomogram, age is a high-risk factor. CSCC is more common in areas where the eyes are exposed to the sun, such as the sun-damaged conjunctiva of the limbus. Therefore, UV rays may be the principal cause of CSCC [26, 27]. With aging, the time that the eyes are exposed to the sun does not accumulate for a short period of time. Old patients have a lower awareness of medical treatment, and the time loss for early treatment is an important a major reason for poor prognosis and increased disease burden. The prognosis for male patients is poorer than for female individuals. Abt et al. and Emmanuel et al. pointed out that male gender is a high-risk factor [28, 29]. In addition to their physiological factors, males spend longer time outdoors than females and thus have longer exposure to UV radiation, which may also be a contributing element of this phenomenon. Although laterality had the least impact on the prognosis of patients with CSCC in the new model, the prognosis of tumors in the left eye is still worse than that in the right eye. Previous research explanations have been proposed for the laterality imbalance, including the differing routes of blood supply to both eyes or an asymmetric effect of reading saccades. The present results revealed that tumor N2 and MX had a worse prognosis in patients with CSCC than N1 and M0, respectively. The main reason is that further lymph node metastasis occurs at N2 and MX stages (although MX cannot be determined as a distant metastasis site, its possibility of distant metastasis is greater than M0). T staging has no influence according to the multivariate analysis. However, Bellerive et al. pointed out that the AJCC staging of CSCC is not a reliable guide for initial treatment. The fundamental reason is that T staging is inaccurate, and the reclassified T3 category (diffuse and deep infiltration) can effectively guide the patient's initial treatment [12]. In the new model, a high grade, low differentiation of tumor cells, and high degree of tumor malignancy indicate poor patient prognosis. This finding is consistent with the conventional clinical situation. Nagarajan et al.'s findings demonstrate that PD-L1 is expressed in almost half of CSCC, The density of tumor-associated immune cells correlated with invasive CSCC, stage in CSCC [30]. Surgery is a protective factor in the nomogram, and surgical treatment (including intraorbital resection) is the significant choice for advanced CSCC. Compared with that of early diseases, the recurrence of advanced tumors after resection is more frequent [31]. Therefore, patients with CSCC should be identified and treated as soon as possible. Chemotherapeutic drugs such as mitomycin C, interferon-*α*2b, and 5-fluorouracil have been highly recognized and accepted, and drug treatment has grown popular. [32]. An initial case series has described that pure local chemotherapy without surgery is safe, effective, and can completely resolve ocular surface squamous tumors [33]. According to the established nomogram, as long as the patient's information may be used to determine the score corresponding to the variable, the survival probability of the patient in the corresponding year is the total score obtained after the addition corresponds to the scale of the survival probability line of 3, 5, and 8 years below the total point line.

## 5. Conclusions

Six risk factors, namely, age, sex, grade, laterality, N, M, and surgery were explored and integrated into a model to establish a nomogram, which was then verified through multiple perspectives of discrimination, calibration, improvement, and clinical decision-making benefits. The model was proven to be trustworthy and accurate in its predictions. Compared with the current AJCC (TNM) that fails to provide high-quality guidance in the treatment and prognosis of CSCC (limited to patients), the proposed model may accurately estimate the survival rate of patients with CSCC through patient information. This is the first study to establish a prognostic nomogram for CSCC, this tool allows clinicians to provide effective guidance during decision-making.

## 6. Limitations

This is a retrospective study, and there will inevitably be biases. Our data comes from the SEER database, and the promotion of conclusions is limited. Owing to the limited public information provided by the database and the lack of laboratory data, only a few factors were included in this study. Regardless, this research is meaningful and can provide a reliable reference for clinicians and patients.

## Figures and Tables

**Figure 1:** E.g., only small lesions can be completely removed, and large lesions involving the orbit may require orbital exenteration.

**Figure 2:** Flowchart of the research.

**Figure 3:** Nomogram of conjunctival squamous cell carcinoma.

**Figure 4:** ROC curves between the nomogram and the TNM staging system, training set (a, b, c), validation set (d, e, f).

**Figure 5:** Calibration curve at 3, 5, and 8 years, training set (a, b, c), validation set (d, e, f).

**Figure 6:** DCA curves for the 3, 5, and 8 years, training set (a), validation set (b).

**Table 1:** Baseline characteristics of patients.

Variable	Train			Test		
	Alive (324)	Dead (196)	*P* value	Alive (77)	Dead (53)	*P* value
Age	62 [51-71]	77 [69-84]	<0.001	62 [53-70]	77 [64-84]	<0.001
Sex			0.008			0.633
Male	224 (69.1)	157 (80.1)		57 (74)	42 (79.2)	
Female	100 (30.9)	39 (19.9)		20 (26)	11 (79.2)	
Grade			0.011			0.083
I	78 (24.1)	43 (21.9)		22 (28.6)	11 (20.8)	
II	46 (14.2)	38 (19.4)		16 (20.8)	7 (13.2)	
III	13 (4.0)	18 (9.2)		1 (1.3)	5 (9.4)	
IV	0 (0.0)	2 (1.0)		2 (2.6)	0 (0.0)	
Unknown	187 (57.7)	95 (48.5)		36 (46.8)	30 (56.6)	
Laterality			0.772			0.823
Left	155 (47.8)	100 (51.0)		36 (46.8)	22 (41.5)	
Right	165 (50.9)	94 (48.0)		40 (51.9)	30 (56.6)	
Unknown	4 (1.2)	2 (1.0)		1 (1.3)	1 (1.9)	
Stage			0.816			0.979
Localized	273 (84.3)	161 (82.1)		65 (84.4)	45 (84.9)	
Regional	18 (5.6)	12 (6.1)		4 (5.2)	3 (5.7)	
Unknown	33 (10.2)	23 (11.7)		8 (10.4)	5 (9.4)	
T			0.551			0.25
TX	188 (58.0)	125 (63.8)		40 (51.9)	29 (54.7)	
T1	65 (20.1)	32 (16.3)		20 (26.0)	6 (11.3)	
T2	28 (8.6)	17 (8.7)		9 (11.7)	8 (15.1)	
T3	36 (11.1)	16 (8.2)		6 (7.8)	2 (3.8)	
T4	7 (2.2)	6 (3.1)		2 (2.6)	29 (54.7)	
N			0.369			0.34
N1	45 (13.9)	25 (12.8)		11 (14.3)	4 (7.5)	
N2	276 (85.2)	171 (87.2)		65 (84.4)	49 (92.5)	
N3	3 (0.9)	0 (0.0)		1 (1.3)	0 (0.0)	
M			0.448			0.528
M0	291 (89.8)	171 (87.2)		69 (89.6)	50 (94.3)	
MX	33 (10.2)	25 (12.8)		8 (10.4)	3 (5.7)	
Surgery			0.528			0.529
Yes	279 (86.1)	164 (83.7)		64 (83.1)	47 (88.7)	
No/unknown	45 (13.9)	32 (16.3)		13 (16.9)	6 (11.3)	
Race			0.001			0.109
Black	12 (3.7)	6 (3.1)		2 (2.6)	3 (5.7)	
Other	38 (11.7)	5 (2.6)		11 (14.3)	2 (3.8)	
White	274 (84.6)	185 (94.4)		64 (83.1)	48 (90.6)	

**Table 2:** Multifactor COX analysis results.

Variable	Multivariable analysis		*P* value
	HR	95% CI	
Age	1.077	1.061-1.093	<0.001
Sex			
Male	Reference		
Female	0.691	0.480-0.994	0.046
Grade			
I	Reference		
II	0.925	0.590-1.453	0.737
III	1.069	0.586-1.950	0.828
IV	7.857	1.651-37.391	0.010
Unknown	0.823	0.567-1.195	0.306
Laterality			
Right	Reference		
Left	1.403	1.049-1.875	0.022
Unknown	1.122	0.249-5.053	0.881
N			
N1	Reference		
N2	7.195	1.560-33.191	0.011
N3	<0.001	0	0.993
M			
MX	Reference		
M0	0.217	0.049-0.961	0.044
Surgery			
Yes	Reference		
No/unknown	1.618	1.006-2.601	0.047

**Table 3:** NRI and IDI values of the model.

	IDI				NRI			
	train	P	test	P	train	lower-upper	test	lower-upper
3-Year	0.122	P<0.001	0.095	P<0.001	0.651	0.404-0.934	0.629	0.142-1.025
5-Year	0.209	P<0.001	0.175	P<0.001	0.768	0.518-0.953	0.771	0.328-1.101
9-Year	0.263	P<0.001	0.226	P<0.001	0.802	0.300-1.021	0.675	0.312-1.206

## Data Availability

SEER collects cancer incidence from population-based cancer registries with a data coverage greater than 30% of the U.S. population. The data we used is based on the November 2021 submission. We accessed these through the SEER^∗^Stat software with additional approvals.
